This article has been retracted.

# Safety and Efficacy of Mild Moxibustion on Cancer-Related Fatigue in Non-Small-Cell Lung Cancer Patients Undergoing Chemotherapy

**DOI:** 10.1155/2022/6530454

**Published:** 2022-07-22

**Authors:** Xiaomin Xu, Fen Gu

**Affiliations:** ^1^Department of Nephrological and Cardiovasology, Shanghai Baoshan District Wusong Central Hospital, Shanghai 200940, China; ^2^People's Hospital of Shanghai Putuo District, Shanghai, China; ^3^Nursing Department, Shanghai Ninth People's Hospital, Shanghai Jiaotong University School of Medicine, Shanghai 200011, China

## Abstract

**Objective:**

Cancer-related fatigue (CRF) is a well-recognized issue for cancer patients undergoing chemotherapy; however, research on nonpharmacological alternatives have been underreported. This study is aimed at investigating the effect of mild moxibustion on CRF in patients with non-small-cell lung cancer (NSCLC) undergoing chemotherapy.

**Methods:**

A randomized controlled trial was performed on 126 NSCLC patients undergoing initial chemotherapy and were divided into the following three groups: mild moxibustion group, sham acupoint group, and control group. Moxibustion was performed on two groups of acupuncture points, Dazhui and Geshu acupoints in the prone position and Qihai, Guanyuan, and Zusanli acupoints in the supine position, during the chemotherapy for 30 min with one of the groups of acupuncture points per day. Moxibustion of the sham group was performed 1 cm away from the true acupoint, while only routine nursing care was given to the routine group. The efficacy and safety of the treatments were assessed based on the Chinese version of the Revised Piper Fatigue Scale (RPFS-CV), the quality of life (QoL) questionnaire for Chinese cancer patients receiving chemobiotherapy (QLQ-CCC), and liver and kidney function indexes.

**Results:**

A total of 118 cases completed all interventions. There was no significant difference in the baseline indicators among the three groups of NSCLC patients. Although all three groups demonstrated raised RPFS-CV scores over the chemotherapy cycle, comparatively, the mild moxibustion group had significantly lower RPFS-CV scores and better relief of CRF symptoms (*P* < 0.05). The QLQ-CCC results indicated that the QoL of NSCLC patients dramatically decreased following chemotherapy, even with mild moxibustion. Further, mild moxibustion intervention did not show significantly different levels of alanine aminotransferase (ALT), aspartate aminotransferase (AST), serum creatinine (Scr), and blood urea nitrogen (BUN) compared with the two other groups (*P* > 0.05).

**Conclusion:**

Chemotherapy is accompanied by elevated fatigue scores and decreased life quality in NSCLC patients. Although mild moxibustion intervention could alleviate CRF in the patients and was not associated with any adverse events and liver and kidney toxicity when combined with chemotherapy, it could not improve their QoL.

## 1. Introduction

Lung cancer is the second most common cancer and the leading cause of cancer death worldwide, with approximately 1.8 million deaths [1, 2]. There were an estimated 19.3 million new cancer cases (excluding nonmelanoma skin cancers) and nearly 10 million cancer deaths (excluding 9.9 million nonmelanoma skin cancers) globally in 2020. Non-small-cell lung cancer (NSCLC) accounts for about 85% of lung cancer diagnoses [3]. Patients with stages IIb to III lung adenosquamous carcinoma (ASC) are often given platinum-based dual-drug chemotherapy [3] to terminate cancer cell division and inhibit cancer DNA synthesis [4–6]. However, these treatments simultaneously damage normal DNA, thereby increasing the risk of gastrointestinal and hematological toxicity [7] and eventually causing fatigue.

Cancer-related fatigue (CRF) is among the most common subjective adverse event associated with chemotherapy, is estimated to affect 80%-96% of NSCLC patients [8], and is difficult to manage [9]. It is characterized by multidimensional symptoms affecting the patients' daily, social, family, and work life and often result in decreased appetite, altered emotional state, and poor treatment responses [10]. CRF has been observed in almost all cancer patients undergoing chemotherapy [11–14]. However, despite ongoing efforts and research in addressing this issue, the CRF mechanism remains unclear, and there is no evidence for the existence of specific intervention drugs, and nonpharmacological methods currently used for CRF alleviation remain challenging [15, 16].

Presently, an increasing number of patients and physicians prefer complementary and alternative medicine (CAM) to control the symptoms of chemotherapy patients and improve their quality of life [17]. As a member of CAM, moxibustion can mobilize the circulation of qi and blood and warmly invigorate yang with the combined actions of firepower and medicinal power on the meridians and acupoints, thereby ascending yang and relieving prostration. As a traditional Chinese medicine (TCM) nursing technique, moxibustion has the advantages of being simple, convenient, and cost-saving. W. Li and L. Li [18] reported that moxibustion combined with 5-hydroxy tryptamine (5-HT) receptor antagonist significantly decreased the rates and degrees of nausea and vomiting due to chemotherapy in lung cancer patients and were superior to simple 5-HT receptor antagonist without apparent adverse reactions. The beneficial effects of moxibustion were demonstrated in various cancers [19, 20]. Compared with other moxibustion methods, mild moxibustion is featured by a high similarity between its effect of warming and invigorating yang and the tonifying principle of CRF in chemotherapy patients with qi deficiency and yang deficiency. However, there is a lack of randomized clinical trials on the efficacy and QoL of mild moxibustion in NSCLC lung cancer patients undergoing chemotherapy.

This study used mild moxibustion to determine its potential effects on alleviating CRF and improving the quality of life (QoL) of NSCLC patients undergoing chemotherapy to provide clinical evidence for its clinical application in this setting.

## 2. Materials and Methods

### 2.1. Ethics Statement

This randomized clinical trial was approved by the Medical Ethics Committee (201815) of Shanghai Baoshan District Wusong Central Hospital. The patients and caregivers were informed of this study's research purpose, process, and precautions and provided signed informed consent. During the study, the patients were informed that the moxibustion treatment would not affect their anticancer treatment and was aimed at alleviating their discomforts during chemotherapy. The principle of confidentiality was strictly followed without disclosing any personal information associated with the patients, which were only used for academic research purposes. The patients were allowed to withdraw from the trial without giving any reason.

### 2.2. Research Subjects

A total of 126 patients with stage Ib-IIIa NSCLC admitted to three areas of the TCM oncology department, People's Hospital of Shanghai Putuo District, from October 2019 to February 2020, were enrolled in this study. All patients were treated with chemotherapy. According to the body surface area, gemcitabine 1,000 mg/m^2^ was used on the 1st and 8th day, and 120 mg/m^2^ of cisplatin was given on the chemotherapy days 1, 2 and 3 and rested for the remaining days. The treatment course was 8 days, and 21 days represented on chemotherapy cycle.

#### 2.2.1. Diagnostic Criteria

NSCLC was diagnosed based on the following criteria: (1) pathological or cytological diagnosis, (2) staging diagnosis of NSCLC according to the 8th edition of International Association for the Study of Lung Cancer (IASLC) TNM staging, and (3) TCM syndrome types were diagnosed according to the Shanghai Traditional Chinese Medicine Diagnosis and Treatment Convention (2nd edition). Consumptive disease was presented as yang deficiency and qi deficiency alone or together.

#### 2.2.2. Inclusion Criteria

The inclusion criteria were as follows: (1) patients diagnosed with NSCLC referred to the diagnostic criteria above; (2) 18-80 years old; (3) patients who were about to undergo the first GP chemotherapy, with an 8-day course of treatment (day 1-3 days and 8); (4) no history of surgery within 6 months before chemotherapy; (5) patients who never participated in any fatigue-related interventions; (6) no infection, injury, and ulcer around the acupoints; (7) patients were diagnosed CRF in line with the CRF diagnostic criteria of the 10th edition of the International Statistical Classification of Diseases and Related Health Problems and were rated as mild and moderate fatigue according to the Chinese version of the Piper Fatigue Scale-Revised (RPFS-CV); (8) had a Karnofsky (KPS) efficacy status score > 60 points, with a predicted survival time > 6 months; (9) no cognitive impairment; and (10) voluntarily participated in this study and provided signed informed consent.

#### 2.2.3. Exclusion Criteria

The exclusion criteria are as follows: (1) consumptive disease syndrome types of lung-kidney yin deficiency and liver-kidney yin deficiency; (2) cancer metastasis; (3) hemorrhagic disease or severe organ dysfunction; (4) diabetes and other sensory disturbances; (5) allergy to moxibustion and skin damage; (6) mental illness; and (7) pregnant women.

#### 2.2.4. Rejection Criteria

Following the start of the study, patients were rejected if (1) their chemotherapy regimen was changed during the study; (2) other treatment regimens were added, i.e., radiotherapy, intervention, and targeted therapy; (3) severe changes in condition and/or termination of chemotherapy during the study; (4) abnormal coagulation indexes and even bleeding during the study; (5) severe fatigue during the study.

#### 2.2.5. Dropout Criteria

The dropout criteria are as follows: (1) patients requested to withdraw during the study and (2) patients with incomplete data or lost to follow-up.

### 2.3. Patient Grouping

According to the above inclusion and exclusion criteria, various indicators of NSCLC patients were evaluated and screened. The patients were numbered by a computer and randomly assigned to three groups (control group, mild moxibustion group, and sham acupoint group), with 42 patients in each group. In addition, the TCM oncology groups in three wards of the TCM department, after training the medical staffs, were responsible for diagnosis, treatment, and using a similar model of nursing.

### 2.4. Routine Nursing and GP Chemotherapy

#### 2.4.1. Chemotherapy-Related Nursing

100 ml of gemcitabine was infused within 30 minutes to avoid drug toxicity. After that, we observed whether the patients had rash, cough, or flu-like symptoms and were informed of the possible symptoms. Besides, the infusion of 500 ml of cisplatin was completed within 2 hours using light-proof leather strips and light-proof bags. After administration, 3000 ml of liquid (intravenous and oral) for hydration, a diuretic was injected to protect renal function with frequent observations of the color, quality, and quantity of the patient's urine. The physician was notified if there was any abnormality. In addition to chemotherapy drugs, antiemetic and gastric protective drugs were simultaneously given as protective measures. Moreover, the patient's blood biochemical index report was observed, and guidance was given to the patient and caregivers about the potential condition associated with changes in the main indexes. The patients were also guided to self-observe their indexes.

#### 2.4.2. Infusion Catheter Care

In principle, chemotherapy drugs are infused using a central venous catheter, peripherally inserted central venous catheter (PICC), and implantable venous access port. In this study, 120 of the 126 patients were administered chemotherapy through a PICC and 6 patients through a superficial vein indwelling needle for personal reasons. After PICC placement, the dressing was changed once within 24 hours. Besides, patients were informed not to bend, straighten, and raise the arm on the side of the catheter as much as possible within 3 days. After 3 days of catheter placement, the patients could perform normal daily work. The PICC was maintained once a week during the treatment period. Further, attention was paid to measuring the arm circumference of the patient's puncture side, observing the local skin condition of the puncture point, and adjusting the catheter length. Afterward, the catheter was flushed and sealed properly with the condition recorded. Before and after infusion of chemotherapeutic drugs with a superficial vein indwelling needle, a 20 ml sterile syringe was used to aspirate normal saline to flush the tube. During the infusion, the local skin condition was strictly observed. If there was redness and swelling, the needle was pulled out immediately, and symptomatic treatment was performed depending on the local skin condition and the nature of the chemotherapeutic drug.

#### 2.4.3. Diet Care

During chemotherapy, the patients were advised to consume healthy diets with mainly high-calorie, high-vitamin, easy-to-digest foods, and more green leafy vegetables. Additionally, different dietary guidance was provided depending on the patient's TCM syndrome type. For example, patients with lung-spleen qi deficiency were guided to eat atractylodes poria and white fungus porridge, those with heart-spleen deficiency were advised to eat astragalus and codonopsis chicken soup, those with lung-kidney yang deficiency to eat yam and black chicken porridge, and those with heart-kidney yang deficiency to eat yam and chestnut porridge.

#### 2.4.4. Emotional Care

According to the attributes of TCM for lung diseases, the patients were guided to listen to Shang-tuned music, such as *Your Legend, Fifteen of the moon and Symphony No.3*, while undergoing psychological care (patient explanation and encouragement), with the intention to balance their thoughts, remain calm, and purify and send lung qi.

#### 2.4.5. Exercise Guidance

During chemotherapy, the patients were asked to do exercises such as Twelve Chapter Brocade, breathing exercises, and yoga meditation. If their fatigue worsened, they were advised to save physical strength and the exercise was modified depending on their condition.

#### 2.4.6. Guidance for Follow-Up Visits

Before discharge, the patients were instructed for regular follow-up visits and given a guidebook on CRF and a daily management record book. On the day of the follow-up visit, the contents of the patients' record book were checked and queried on their daily management, and any questions were answered in time. If the patient revisited at the nearest community hospital, they were followed up by telephone on the same day evening, and their blood biochemical examination data were recorded and guided on daily management.

### 2.5. Group Intervention

The patients were grouped into a control group, mild moxibustion group, and sham acupoint group. Patients from the control group were only treated with routine nursing and chemotherapy. In the mild moxibustion group, the patients received mild moxibustion intervention, routine nursing, and chemotherapy. In the sham acupoint group, in addition to routine nursing and chemotherapy, moxibustion was performed at a sham acupoint 1 cm far away from the true acupoints of the mild moxibustion group. Other operations were the same as those in the mild moxibustion group. The intervention regimen of moxibustion included two sets of acupoints, with one set performed per day: Dazhui and Geshu acupoints in the prone position and Qihai, Guanyuan, and Zusanli acupoints in the supine position. According to the yang principle before yin, moxibustion was performed in the prone position on the first day. The above acupoints were determined following the *Meridian and Acupoint Science*, a “Thirteenth Five-Year Plan” textbook for higher education on TCM in China. The acupoints were named and located as follows: (1) Dazhui (GV14): in the depression below the spinous process of the 7th cervical vertebra, on the posterior midline; (2) Geshu (BL17): below the spinous process of the 7th thoracic vertebra, 1.5 inches lateral to the posterior midline; (3) Qihai (CV6): 1.5 inches below the umbilicus, on the anterior midline; (4) Guanyuan (CV4): 3 inches below the umbilicus, on the front midline; and (5) Zusanli (ST36): 3 inches below Dubi, on the line connecting Dubi and Xiexi. The specific operations are illustrated as follows. Firstly, the Happyall moxibustion, 5-year-old moxa sticks (diameter: 15 mm and height: 22 mm), and tape (diameter of the middle circular hole: 4 cm) were purchased from the Chongqing Happyall Medical Equipment Co., Ltd. Then, the tape was put into the moxibustion tube (diameter: 39 mm and height with the cover: 63 mm). After peeling off the backing paper, it was stuck on the moxibustion acupoint with the moxibustion cover removed. The moxibustion sticks were completely and sequentially inserted into the socket of the moxibustion cover following ignition. After the fire was self-extinguished, the cover was put into the moxibustion cylinder, and the air outlet size was adjusted to half, which was 3 cm away from the skin. During moxibustion, the patient was maintained at a suitable temperature by adjusting the temperature of moxibustion, such as raising the adjusting cylinder and rotating the moxibustion cover to adjust the size of the air outlet. In this study, the patients were administered a treatment course of 12 days when their conditions were observed. They received mild moxibustion intervention in the morning routine nursing time on the day of chemotherapy, once a day for 30 minutes. Besides, the intervention continued until the 4th day after chemotherapy, for 12 days. Additionally, there were no differences between the sham acupoint group and the mild moxibustion group except for the moxibustion location (sham acupoints 1 cm next to the true acupoints). The patient's fatigue numerical rating scale scores, local skin conditions, tongue, coating, pulse, and syndrome types were recorded every day before the intervention.

### 2.6. Quality Control

Before the intervention, the medical staff were trained in the theoretical operation and listened to the patients' feelings. After passing the assessment, they entered the intervention stage. During the intervention, the following operations were performed to avoid mistakes: (1) a detailed assessment of the patient was conducted before each moxibustion; (2) a physician was present to supervise the moxibustion; (3) for hospitalized patients, the researchers uniformly sent out the material and had patients answered all questions on the spot. If there were any missing items, the patient was asked to complete them in time; (4) before discharge, the researcher established a WeChat group to answer questions and collect data. Patients without WeChat were contacted by phone; (5) all data were entered by two persons. If there is any inconsistency, corrections were made after checking.

### 2.7. Prevention and Treatment of Adverse Reactions

#### 2.7.1. Dizzy Moxibustion

Dizzy moxibustion is uncommon and could be prevented by some precautionary steps. For first-time moxibustion patients, they were informed about the procedure in advance to make them relax and calm during the moxibustion process. Before each moxibustion, the patient's physical and mental health was assessed. During moxibustion, the patients' conditions were observed, asked about any discomforts, and inquired about chief complaints. After the moxibustion, the patients were assisted to sit up slowly for 10 min in the waiting area and were allowed to leave after confirming the absence of any discomforts to avoid delayed dizzy moxibustion effects. However, if the patients experienced dizziness, cold sweat, chest tightness, and palpitation, corresponding treatments were offered in time. In mild cases, it was advised to place the patients in a supine position, and their collar was untied. The patient was then instructed to relax, guided to take a deep breath, and drink warm water. Nevertheless, if the patients suddenly lost consciousness and their face turned gray, the doctor was urgently notified, venous access was simultaneously opened, an electrocardiogram (ECG) monitor was connected, and an ambulance was rushed to the bedside for backup.

#### 2.7.2. Moxibustion Blister

Prevention: generally, mild moxibustion does not cause moxibustion blisters, and the slightly red skin surface after moxibustion is a normal phenomenon. Before moxibustion, an assessment was performed on the patient. During moxibustion, the patient's emotions and feelings were inquired. After moxibustion, the local skin of the patient was observed. Treatment: patients with moxibustion blister(s) were treated differently depending on the size of the blister. Patients with small blister(s) were told that the moxibustion blister would be self-absorbed and advised to irritate or rub the surface of the skin. Those with larger blister(s) were suctioned with a sterile syringe and then sterilized again. Besides, the patients were told not to tear off the surface of the moxibustion blister to avoid infection. Moreover, they were informed to take a bath on the limbs where the moxibustion blisters were located. Additionally, moxibustion nurses recorded the time, size, and treatment of moxibustion blisters and reported the nursing adverse event.

#### 2.7.3. Allergies

Prevention: the patients' conditions were evaluated before the moxibustion, asked for the presence of any discomforts during the process, and their local skin was observed after moxibustion. Treatment: patients with small-scale erythema rash were instructed not to scratch the area as they would subside on their own. In the cases of systemic symptoms, the patients were given medicine prescribed by the doctor.

### 2.8. Observation Indicators

#### 2.8.1. Main Indicators

The Chinese version of the Revised Piper Fatigue Scale (RPFS-CV) was revised by Hong Kong scholars in 2003 [21]. It was implanted in this study to assess CRF in the patients within 2 hours of admission on the 8th, 12th, and 21st days of chemotherapy. It consisted of 28 items. Compared with the original version, the revised version contained a judgment item before item 1, namely, “Have you felt fatigued recently (in the past 4 weeks)?” If the answer was “No,” there was no need to continue the following questionnaire. In addition, a “not applicable” option was added to the description of sexual life in item 5 of the original scale. For patients who were not sexually active, this option could be ticked. Furthermore, the test-retest reliability and Cronbach alpha coefficient of the RPFS-CV scale in the Chinese population were 0.98 and 0.91, and its four dimensions ranged between 0.89 and 0.93, showing good reliability and validity. In this study, the Cronbach's alpha coefficient of the scale was 0.72, with good internal consistency.

#### 2.8.2. Secondary Indicators

The QoL questionnaire for Chinese cancer patients receiving chemobiotherapy (QLQ-CCC) was completed within 2 hours of admission on the 8th and 21st days of chemotherapy [22]. This scale was compiled by Luo et al. [22] in the 1990s and is suitable for all cancer and cancer treatment patients. Besides, the scale contains 35 items involving 5 dimensions: physical, psychological, social, disease, and other items. It adopts Likert 5-level for scoring, while items 1, 4, 5, 7, 9, 10, 13, 14, 17, 18, 20, 21, 22, 24, 27, 28, and 30 were for reverse scoring. Moreover, the higher the QLQ-CCC scores, the better the patient's QoL. In addition, the Cronbach alpha coefficient of QLQ-CCC in cancer patients was 0.925, and in this study, it was 0.80.

#### 2.8.3. Security Indicators

The incidence of mild moxibustion side effects was evaluated by observing the appearance of dizzy moxibustion, moxibustion blisters, and allergic adverse reactions after daily moxibustion. Specifically, routine blood samples were collected from the patients within 2 hours of admission on the 8th, 11th, and 21st days of chemotherapy. Then, the collected samples were sent to the outpatient testing center for testing and to evaluate the liver and kidney functions.

### 2.9. Statistical Analysis

All data were analyzed using the Statistical Package for Social Sciences (SPSS) v19.0 software. If the baseline data of the patients conformed to a normal distribution with homogeneous variance, the measurement data (age, course of disease, scale scores of continuous variables, and various blood indexes) were expressed as *χ* ± *s* and analyzed with the one-way analysis of variance (measurement data). However, if it does not meet the normal distribution and/or has an uneven variance, different methods, such as logarithmic conversion, were firstly selected to perform a normal conversion according to the degree of skewness. If the situation remained unsatisfactory, it was expressed as the median, the Kruskal-Wallis H test was used for K independent samples, and count data (gender, education, etc.) were expressed as frequency and percentage. The chi-square test was performed when the theoretical frequency was ≥5, and the Fisher's exact test was applied if the theoretical frequency was ≤5. If the scores of the RPFS-CV and QLQ-CCC conformed to a normal distribution with homogeneous variance, repeated variance measures were used for analysis. When the spherical test had a *P* value > 0.05, the results of the within-subject effect test were observed, and the multivariate test results were observed when *P* < 0.05. Analysis of variance was measured repeatedly, and a simple effect analysis was required if the results showed an interaction between groups and time. Further pairwise comparisons were performed if the results did not show interaction, and the main effect was *P* < 0.05. Transformation was first performed if it did not conform to the normal distribution and/or homogeneity of variance. If the situation remained unsatisfactory, the generalized estimating equation was used to analyze and test the results.

## 3. Results

### 3.1. Research Objects

In the early stage of this study, a total of 126 eligible NSCLC patients were included and randomly divided into 3 groups, with 42 patients in each group. Of these patients, 2 in the mild moxibustion group had severe fatigue and stopped the intervention. In the sham acupoint group, 1 patient terminated the chemotherapy due to intolerance, 1 patient was transferred to another hospital midway through the intervention, and 1 patient had severe fatigue and stopped the intervention. In the control group, 1 patient changed the chemotherapy regimen, and 2 suspended the chemotherapy midway due to the severe decline in leukocyte levels. Therefore, 118 cases with complete data were finally intervened, including 40 cases in the mild moxibustion group, 39 cases in the sham acupoint group, and 39 cases in the control group. The grouping process of the selected patients is shown in Figure 1.

### 3.2. General Information

The baseline data of the 118 included NSCLC patients are shown in Table 1. The table shows no significant difference in general baseline data among the three groups (control group, mild moxibustion group, and sham acupoint group). The general baseline data included age of NSCLC patients, CRF score, patient quality of life score after chemotherapy, KPS efficacy status score, alanine aminotransferase (ALT) level, aspartate aminotransferase (AST) level, creatinine (Scr) level, blood urea nitrogen (BUN) level, gender, marriage, education, occupation, disease course, cancer stage, and TCM syndrome type (*P* > 0.05). The above suggested that before the intervention, patients in each group had similar clinical characteristics, chemotherapy functional status, fatigue status, quality of life, and liver and kidney function, allowing further intervention research.

### 3.3. Effect of Mild Moxibustion on RPFS-CV Score of NSCLC Patients during Chemotherapy Cycle

To clarify the relieving effect of mild moxibustion on CRF during the chemotherapy cycle, we evaluated the fatigue status of NSCLC patients in each group using the RPFS-CV. The results showed that the RPFS-CV scores of the three groups of patients conformed to the spherical test (*P* > 0.05) and were normally distributed with homogeneous variance.  Table 2 and Figure 2 show that the results of the within-subject effect test indicated no interaction with fatigue among the three groups, and only the main effects of the intervention method and time needed to be analyzed. Compared with the sham acupoint and control groups, the mild moxibustion group presented a lower RPFS-CV score (*P* < 0.05), while there was no statistical difference in the RPFS-CV score between the sham acupoint and control groups. In addition, it was also found that the RPFS-CV scores of patients in each group on the 8th, 12th, and 21st days of chemotherapy were significantly increased compared with 1 day before chemotherapy. Moreover, with the prolongation of the chemotherapy cycle, the RPFS-CV scores of the patients in each group kept rising. The above suggested that the RPFS-CV scores of NSCLC patients in each group increased over the chemotherapy cycle. Mild moxibustion intervention could significantly reduce the RPFS-CV scores of chemotherapy NSCLC patients and relieve CRF symptoms.

### 3.4. Effects of Mild Moxibustion on the QLQ-CCC Scores of NSCLC Patients during Chemotherapy

To further investigate whether mild moxibustion impacted the QoL of NSCLC patients during chemotherapy, QLQ-CCC was used to assess their QoL 1 day before chemotherapy (T1) and the 8th and 21st days of chemotherapy. According to statistical analysis, the QLQ-CCC scores of the three groups of patients were in line with normal distribution and homogenous variance as well as the sphere test *P* > 0.05. Using the within-subject effect test (Table 3 and Figure 3), we observed no interaction in the quality of life among the three groups of NSCLC patients without obvious difference in the QLQ-CCC scores of patients in each group in the same chemotherapy cycle. Moreover, the QLQ-CCC scores of patients in each group remarkably decreased on the 8th and 21st days of chemotherapy compared with those on the 1st day before chemotherapy (*P* < 0.01). The above suggested that chemotherapy significantly reduced the QoL of NSCLC patients, while mild moxibustion intervention had no obvious effect on the QoL of patients undergoing chemotherapy.

### 3.5. Effect of Mild Moxibustion on Liver and Kidney Function of Patients and Adverse Reactions during Chemotherapy Cycle

Here, we measured the level of liver and kidney function indicators in each group of NSCLC patients during the chemotherapy cycle, such as ALT, AST, Scr, and BUN. According to the statistical results in Table 4, there was no remarkable difference in the ALT, AST, Scr, and BUN levels among the NSCLC patients in each group (*P* > 0.05). Besides, no significant difference was observed in the above indicators with the prolongation of the chemotherapy cycle (*P* > 0.05). Similarly, there was no interaction between liver and kidney functions of the three groups of NSCLC patients. The above evidence indicated that mild moxibustion intervention hardly improved the liver and kidney functions of NSCLC patients during chemotherapy. Of note, the patients did not have adverse reactions, such as dizzy moxibustion, moxibustion blister, and allergy, during the whole intervention process.

## 4. Discussion

In this study, acupoints were selected from three meridians: the Zusanli point of the stomach meridian of the Foot-Yangming, the Qihai and Guanyuan point of the Ren channel, and the Dazhui and Geshu of the Du channel. They are all specific acupoints, and the intervention was performed following the meridian qi's different confluence and operation modes. Such acupoints are the most widely used clinically with many indications. Studies have reported that platinum-based chemotherapy could impair gastric motility in rats, leading to imbalance [23]. Besides, Zusanli acupoint can be stimulated to alleviate the injury of Cajal interstitial cells in the gastrointestinal tract of rats, thereby improving gastric motility and immune function [24]. The study by Guo et al. pointed out that Shenque, Zhongwan, Neiguan, etc., often served as combined acupoints of Zusanli and played a coordinating role in intervening chemotherapy drugs to improve nausea and vomiting [25]. In addition, moxibustion at Zusanli could effectively upregulate the level of white blood cells in mice after chemotherapy. To clarify, the Notch signaling pathway may be activated by regulating CSL, Jagged1, and Notch1. Then, the bone marrow hematopoietic function was enhanced to regulate the corresponding hematopoietic stem cells and relieve fatigue. Guanyuan and Qihai belong to the Ren channel. Guanyuan, also known as Sanjiao, as the name suggests, is the intersection of the three yin meridians of the foot and the Ren channel. Besides, as the small intestine front-mu point, Guanyuan can treat consumptive exhaustion and coldness, thinness, and weakness. A research study reported that moxibustion on Guanyuan point could increase CD3+, CD4+, CD4+/CD8+, and NK cells in cancer patients [26], and this acupoint could also be stimulated to reduce serum IL-6 and TNF-*α* in rats and inhibited the apoptosis of thymocytes and spleen cells [27]. From the above, we found that the intervention of Guanyuan acupoint might strengthen immune function, reduce inflammatory responses, stabilize and gradually improve the righteousness in the body, and relieve\fatigue. As the original point of man, Qihai is located above Guan Yuan and is also known as Xia Man. By stimulating the Qihai acupoint, the average cell value can be remarkably increased in patients with CRF and improve fatigue symptoms [28]. Usually, the Guanyuan point and Qihai point are combined to achieve a multiplier effect. According to the experiments and clinical studies of Lin Yumin [29], moxibustion on Qihai and Guanyuan could increase the level of IgG and IgM in fatigued rats, reducing fatigue scores rating scale and anxiety self-rating scale of patients. As for Geshu and Dazhui, they are both located on the back of the human body. Studies have shown that mild moxibustion intervention could effectively relieve bone marrow suppression and elevate white blood cell counts in chemotherapy-treated mice. Compared with acupuncture, moxibustion was more conducive to antagonizing the damage of hematopoietic progenitor cells caused by inhibitory regulators [30]. The Dazhui acupoint, also known as Bailao, belongs to the Du channel. It is located at the intersection of the six yang meridians and the Du channel. Considering the effect of controlling all yang qi, Dazhui is regarded as yang within yangi. Studies have indicated multiple pathways for regulating the mechanism of moxibustion on cancer remission [31]. Moreover, moxibustion at the Dazhui acupoint was found to inhibit tumor necrosis and hemorrhage. Tan Li et al. analyzed the point selection rules of moxibustion for bone marrow inhibition after radiotherapy and chemotherapy [32]. In this study, we found that the meridians mainly referred to the Du meridian and bladder meridian, with a commonly used combination acupoint of shu-back as Dazhui, Zusanli, and Geshu were the most frequently used. Ma et al. summarized the effect of moxibustion intervention on patients' symptoms during chemotherapy and showed that moxibustion could regulate the immune function of patients, relieve bone marrow suppression, improve the degree of CRF and improve QoL [33].

In addition, the results of Oh and Cho [34] revealed that from the start of the first cycle of chemotherapy to the start of the next cycle of chemotherapy, the patient's fatigue level increased over time regardless of the intervention method. Through follow-up, we found the persistence of such an upward trend in fatigue until all chemotherapy cycles were completed. The reasons for the above results may be responsible for the accumulation of chemotherapeutic drugs in the body and the half-life period. Our results also showed that the degree of fatigue in NSCLC patients continued to increase over chemotherapy. Although the degree of fatigue was rising, the increasing trend of fatigue in the mild moxibustion group was significantly slower than in the control and sham acupoint groups, suggesting that mild moxibustion may play a role in relieving fatigue. In addition, according to statistics, within a short time after the first course of chemotherapy, the increase in patient's fatigue slowed down, but the significance between that during chemotherapy did not reach significance, indicating that the symptoms of CRF in cancer patients may be affected and counteracted by a variety of factors in addition to the effect of chemotherapy drugs. Besides, from the later interviews, most patients' nervousness was significantly relieved after the last day of periodic chemotherapy, and descriptions such as “relieved” were mentioned. The above findings suggested that the degree of CRF during chemotherapy could also be related to changes in mood, similar to the research results of He and Wu [35]. Collectively positive psychology could reduce the negative emotions of patients undergoing chemotherapy and thus reduce the degree of fatigue.

This study revealed that mild moxibustion intervention could not remarkably improve the QoL of NSCLC patients undergoing first-time chemotherapy. According to the trend chart, the quality of life of NSCLC patients declined with chemotherapy. However, it remained relatively stable rather than declined from the end of chemotherapy to the beginning of the next chemotherapy cycle. This finding was inconsistent with most studies [36–39]. We hypothesize that there could be three reasons for such observation: the moxibustion type, intervention course of treatment, and rating scale type. At present, thunder-fire moxibustion or grain moxibustion embodies the most obvious effect on moxibustion intervention for patients with lung cancer undergoing chemotherapy. Similar to mild moxibustion, thunder-fire moxibustion belongs to the category of suspended moxibustion but with a much larger diameter than the moxa stick. Wang et al. [40] reported that the temperature of thunder fire after burning was higher than that of mild moxibustion. The effects of thunder-fire moxibustion intervention may be enhanced by a larger burning area and higher burning temperature. As for the grain moxibustion, it belongs to direct moxibustion and is only protected by a layer of vaseline from the skin during moxibustion, with a high stimulation to the skin. Zhang et al. found that with antioxidant and anti-inflammatory activity, the strong stimulation of grain moxibustion rapidly activated certain conduction pathways in the metabolomics, thereby improving the QoL [41].

Regarding intervention courses, moxibustion may improve the curative effect but usually require long-term intervention. This study considered many influencing factors after the patient was discharged from the hospital. For example, the TCM syndrome differentiation could not be completed in time. Therefore, a continuous intervention was not carried out, which may affect the intervention effect. As for scale selection, the final evaluation results may be affected by multiple types of QoL scales for cancer patients, different evaluators (self-evaluation and other evaluations), differences in content dimensions, and cultural diversity. In addition, QoL cannot be changed by a single factor in a short time. The changes in QoL of cancer patients may be more closely related to disease stages or stages of treatment [42], which may be responsible for the ineffectiveness of mild moxibustion interventions.

The safety of mild moxibustion can be mainly judged from two aspects: the occurrence of adverse events and liver and kidney function. In this study, no patient suffered from adverse events such as dizzy moxibustion, allergy, and moxibustion blisters, which could be attributed to the professional operation of nurses and the relatively mild moxibustion performance. Additionally, ALT, AST, Scr, and BUN were used to evaluate the liver and kidney functions of patients. The statistical results showed no significant difference in the liver and kidney function of the three groups of patients. The above evidence suggests that the mild moxibustion intervention did not exert such effects on the liver and kidney function of the patients compared with chemotherapy drugs. Thus, mild moxibustion had certain safety at the level of blood biochemical indicators.

## 5. Conclusion

In conclusion, mild moxibustion was found to play a significant role in reducing CRF in NSCLC patients undergoing GP chemotherapy and was not associated with any adverse events. The relief effect of CRF could be enhanced by prolonging the intervention time, continuing nursing, and constructing a learning platform for moxibustion intervention. However, it did not improve the patients' QoL compared to the sham and control groups. These findings indicate the potential use of mild moxibustion in diverse settings such as inpatient routine care and home care.

## Figures and Tables

**Figure 1:** Flow chart of the grouping of selected patients.

**Figure 2:** Trend chart of fatigue scores in three groups of NSCLC patients.

**Figure 3:** Trend chart of QLQ-CCC scores in three groups of NSCLC patients.

**Table 1:** General clinical data.

Variable	Control group (*n* = 39)	Sham acupoint group (*n* = 39)	Mild moxibustion group (*n* = 40)	*F*/*χ*^2^/*Z*	*P*
Age	56.25 ± 9.05	55.91 ± 7.59	56.62 ± 8.36	0.072	0.930
Disease course	9.95 ± 2.21	9.92 ± 2.03	10.03 ± 2.21	0.024	0.976
RPFS-CV score	1.57 ± 0.73	1.62 ± 0.62	1.55 ± 0.73	0.131	0.877
QLQ-CCC score	126.01 ± 6.37	125.90 ± 6.14	125.20 ± 4.01	0.260	0.773
CRF score	1 (1, 1)	1 (1, 1)	1 (1, 1)	0.222	0.895
KPS score	85.13 ± 5.56	84.87 ± 5.06	84.50 ± 5.04	0.145	0.866
ALT	26.64 ± 10.97	24.53 ± 8.70	24.54 ± 9.74	0.598	0.552
AST	24.07 ± 5.97	24.36 ± 5.70	24.91 ± 6.55	0.194	0.824
SCr	61.07 ± 5.85	62.98 ± 7.33	62.79 ± 8.24	0.833	0.437
BUN	5.11 ± 0.86	5.20 ± 0.75	5.00 ± 0.74	1.014	0.366
Gender					
Male	18 (46.2%)	19 (46.7%)	20 (50%)	0.121	0.941
Female	21 (53.8%)	20 (53.3%)	20 (50%)		
Marriage status					
Unmarried	6 (15.4%)	2 (5.1%)	5 (12.5%)	4.089	0.665
Married	26 (66.7%)	29 (74.4%)	25 (62.5%)		
Widowed	4 (10.3%)	5 (12.8%)	8 (20%)		
Divorced	3 (7.7%)	3 (7.7%)	2 (5%)		
Education					
Primary school	4 (10.3%)	6 (15.4%)	6 (15%)	5.399	0.494
Junior high school	14 (35.9%)	11 (28.2%)	14 (35%)		
Senior high school	16 (41%)	11 (28.2%)	15 (37.5%)		
Undergraduate and above	5 (12.8%)	11 (28.2%)	5 (12.5%)		
Occupation					
Fixed occupation	14 (35.9%)	15 (38.5%)	13 (32.5%)	0.556	0.968
Freelance	5 (12.8%)	4 (10.3%)	6 (15%)		
Retired	20 (51.3%)	20 (51.3%)	21 (52.5%)		
Cancer staging					
Ib	0 (0%)	1 (2.6%)	1 (2.5%)	3.072	1.000
IIa	2 (5.1%)	1 (2.6%)	2 (5%)		
IIb	1 (2.6%)	0 (0%)	1 (2.5%)		
IIIa	36 (92.3%)	37 (94.8%)	36 (90%)		
TCM syndrome type					
Lung-spleen qi deficiency	9 (23.1%)	9 (23.1%)	8 (20%)	2.297	0.890
Dual deficiency of the heart-spleen	11 (28.2%)	14 (35.9%)	15 (37.5%)		
Spleen-kidney yang deficiency	10 (25.6%)	9 (23.1%)	12 (30%)		
Heart-kidney yang deficiency	9 (23.1%)	7 (17.9%)	5 (12.5%)		

RPFS-CV: Chinese version of the Piper Fatigue Scale-Revised; QLQ-CCC: the quality of life questionnaire for Chinese cancer patients receiving chemobiotherapy; ALT: alanine aminotransferase; AST: aspartate aminotransferase; Scr: creatinine; BUN: blood urea nitrogen.

**Table 2:** RPFS-CV scores of three groups of patients.

Group	T1	T8	T12	T21
Control	1.57 ± 0.73	2.16 ± 0.76^a^	2.23 ± 0.77^a^	2.63 ± 0.79^abc^
Mild moxibustion	1.55 ± 0.73	1.74 ± 0.74^∗^^#a^	1.84 ± 0.71^∗^^#a^	2.08 ± 0.83^∗^^#abc^
Sham acupoint	1.62 ± 0.62	2.00 ± 0.73^a^	2.13 ± 0.61^a^	2.49 ± 0.74^abc^

Note: T1: 1 day before chemotherapy; T8: the 8th day of chemotherapy; T12: the 12th day of chemotherapy; T21: the 21st day of chemotherapy. ^a^Difference compared with T1; ^b^difference compared with T8; ^c^difference compared with T21; ^∗^difference compared with the control group; ^#^difference compared with the sham acupoint group.

**Table 3:** QLQ-CCC to assess the QLQ scores of the three groups of patients.

Group	T1	T8	T21
Control	126.01 ± 6.37	117.80 ± 4.17^a^	116.92 ± 2.66^a^
Mild moxibustion	125.20 ± 4.01	119.87 ± 5.52^a^	118.66 ± 3.87^a^
Sham acupoint	125.90 ± 6.14	118.07 ± 4.68^a^	117.52 ± 3.81^a^

Note: T1: 1 day before chemotherapy; T8: the 8th day of chemotherapy; T21: the 21st day of chemotherapy. ^a^There is a difference compared with T1.

**Table 4:** Changes in main liver and kidney function indexes in three groups of NSCLC patients.

Indicators	Between groups		Time		Interaction	
	Wald	*P*	Wald	*P*	Wald	*P*
ALT	3.443	0.196	5.709	0.127	3.022	0.806
AST	0.938	0.625	2.844	0.146	1,925	0.926
Scr	1.197	0.555	2.490	0.477	2.378	0.882
BUN	1.143	0.565	0.072	0.995	4.393	0.624

ALT: alanine aminotransferase; AST: aspartate aminotransferase; Scr: creatinine; BUN: blood urea nitrogen.

## Data Availability

The data used to support the findings of this study are available from the corresponding author upon request.

## Abbreviations

CRF: Cancer-related fatigue
NSCLC: Non-small-cell lung cancer
RPFS-CV: Chinese version of the Revised Piper Fatigue Scale
QoL: Quality of life
QLQ-CCC: QoL questionnaire for Chinese cancer patients receiving chemobiotherapy
ALT: Aminotransferase
AST: Aspartate aminotransferase
Scr: Serum creatinine
BUN: Blood urea nitrogen
ASC: Adenosquamous carcinoma
CAM: Complementary and alternative medicine
TCM: Traditional Chinese medicine
IASLC: International Association for the Study of Lung Cancer
KPS: Karnofsky
PICC: Peripherally inserted central venous catheter
ECG: Electrocardiogram
SPSS: Statistical Package for Social Sciences
Tx: X day
5-HT: 5-Hydroxy tryptamine.
